# Silymarin Targets β-Catenin Signaling in Blocking Migration/Invasion of Human Melanoma Cells

This article has been retracted.

**DOI:** 10.1371/journal.pone.0023000

**Published:** 2011-07-28

**Authors:** Mudit Vaid, Ram Prasad, Qian Sun, Santosh K. Katiyar

**Affiliations:** 1 Department of Dermatology, University of Alabama at Birmingham, Birmingham, Alabama, United States of America; 2 Comprehensive Cancer Center, University of Alabama at Birmingham, Birmingham, Alabama, United States of America; 3 Birmingham VA Medical Center, Birmingham, Alabama, United States of America; University of Pennsylvania School of Medicine, United States of America

## Abstract

Metastatic melanoma is a leading cause of death from skin diseases, and is often associated with activation of Wnt/β-catenin signaling pathway. We have examined the inhibitory effect of silymarin, a plant flavanoid from *Silybum marianum*, on cell migration of metastasis-specific human melanoma cell lines (A375 and Hs294t) and assessed whether Wnt/β-catenin signaling is the target of silymarin. Using an *in vitro* invasion assay, we found that treatment of human melanoma cell lines with silymarin resulted in concentration-dependent inhibition of cell migration, which was associated with accumulation of cytosolic β-catenin, while reducing the nuclear accumulation of β-catenin (i.e., β-catenin inactivation) and reducing the levels of matrix metalloproteinase (MMP) -2 and MMP-9 which are the down-stream targets of β-catenin. Silymarin enhanced: (i) the levels of casein kinase 1α, glycogen synthase kinase-3β and phosphorylated-β-catenin on critical residues Ser^45^, Ser^33/37^ and Thr^41^, and (ii) the binding of β-transducin repeat-containing proteins (β-TrCP) with phospho forms of β-catenin in melanoma cells. These events play important roles in degradation or inactivation of β-catenin. To verify whether β-catenin is a potent molecular target of silymarin, the effect of silymarin was determined on β-catenin-activated (Mel 1241) and β-catenin-inactivated (Mel 1011) melanoma cells. Treatment of Mel 1241 cells with silymarin or FH535, an inhibitor of Wnt/β-catenin pathway, significantly inhibited cell migration of Mel 1241 cells, which was associated with the elevated levels of casein kinase 1α and glycogen synthase kinase-3β, and decreased accumulation of nuclear β-catenin and inhibition of MMP-2 and MMP-9 levels. However, this effect of silymarin and FH535 was not found in Mel 1011 melanoma cells. These results indicate for the first time that silymarin inhibits melanoma cell migration by targeting β-catenin signaling pathway.

## Introduction

Melanoma is the leading cause of death from skin diseases due to its propensity to metastasize. The overall incidence of melanoma is increasing in US, and is increasing rapidly in children. It accounted for an estimated 114,900 new cases of melanoma which were diagnosed in the US for 2010, out of which 68,130 were invasive and resulted in death of nearly 8,700 individuals [1]. Although, melanoma is less common than other types of skin cancer, however, it causes the majority (75%) of skin cancer-related deaths. Activating mutations of the protooncogene *BRAF* have been observed in approximately 50% of malignant melanomas. However, *BRAF* mutations alone are insufficient to cause malignant transformation and other triggering events are needed for melanomagenesis. Once, diagnosed with metastatic melanoma, most patients will ultimately die of their disease within 2 years [2]. Since, melanoma is a highly malignant cancer with a potent capacity to metastasize distantly, an approach that decreases its metastatic ability may facilitate the development of an effective strategy for its treatment and/or prevention.

Phytochemicals offer promising options for the prevention of cancer metastasis. Silymarin is one of them, and this flavanoid is obtained from milk thistle (*Silybum marianum* L. Gaertn.) plant. Silymarin is composed primarily of silibinin (≈90%) together with small amounts of other silibinin stereoisomers, such as isosilybin, dihydrosilybin, silydianin and silychristin [3]. Because silymarin has been shown to have anti-inflammatory, anti-oxidative and anti-carcinogenic effects [4], [5], it has been tested in various *in vitro* and *in vivo* models for its efficacy in prevention of skin carcinogenesis [5]. We previously have shown that topical application of silymarin to sensitive-to-carcinogen (SENCAR) mice resulted in inhibition of 7,12-dimethylbenz(a) anthracene-initiated and 12-O-tetradecanoylphorbol-13-acetate-promoted skin tumorigenesis in terms of tumor incidence, tumor multiplicity and tumor growth [6]. We also have shown that topical application of silymarin inhibits ultraviolet radiation-induced skin carcinogenesis in SKH-1 hairless mice [4]. These studies indicated that silymarin possesses potent anti-skin carcinogenic effects [4]–[6]. Importantly, the chemopreventive effect of silymarin has been studied extensively on non-melanoma skin cancer but its effect on melanoma has not been assessed.

Although the molecular mechanisms underlying the progression of melanoma remain unresolved, various studies have implicated constitutively active Wnt/β-catenin signaling in melanoma progression and metastasis [7], [8]. Non-phosphorylated β-catenin accumulates in the cytoplasm, when activated it enters the nucleus and interacts with T-cell factor transcription factors to control various target genes that are involved in cellular proliferation and migration. Nuclear β-catenin accumulation has been correlated with late stages of tumor progression and metastasis. The presence of mutated β-catenin is associated with aggressive tumor growth and regulates expression of various target genes that mediate cellular processes including proliferation, and migration [9], [10]. In the canonical model of Wnt signaling, β-catenin is phosphorylated at certain key residues by glycogen synthase kinase-3β (GSK-3β) and casein kinase 1 α (CK1α) leading to its ubiquitination and subsequent degradation [11], [12]. Like cancers of other organs, the regulation of β-catenin is lost in melanoma [13]–[15]. This then leads to nuclear accumulation of β-catenin and subsequent stimulation of downstream target genes, which includes the genes of cell proliferation (*e.g.*, cyclins and c-myc) and cell invasion (*e.g.*, matrix metalloproteinases) [16]–[18].

Since metastasis of melanoma is the leading cause of death in humans, in the present study we assessed the chemotherapeutic effects of silymarin on the migration/invasion potential of human melanoma cells. For this purpose, two human metastasis-specific cell lines were selected: A375 which is *BRAF*-mutated and another Hs294t cell line which is also highly metastasis-specific but not *BRAF*-mutated. Normal human epidermal melanocytes were used as a control. In this study we assessed whether silymarin inhibits the migration of melanoma cells and whether it is associated with the inactivation of the β-catenin signaling pathway or decreased accumulation of nuclear β-catenin. In order to verify the role of β-catenin in suppression of melanoma cell migration by silymarin, we compared the effect of silymarin on the behavior of two different melanoma cell lines that differ in their states of constitutive activation of Wnt/β-catenin signaling. The cell lines used were: (a) Mel 1241 cells that are characterized by constitutive activation of β-catenin, and (b) Mel 1011 cells which lack constitutively active β-catenin pathway. Here, we present evidence that silymarin inhibits the invasiveness or migratory potential of melanoma cells by inactivation of β-catenin.

## Materials and Methods

### Cell lines and cell culture conditions

The human melanoma cells lines, A375 and Hs294t, were purchased from the American Type Culture Collection (Manassas, VA), while melanoma cells Mel 1241 and Mel 1011 were a kind gift from Dr. Paul Robbins (Center of Cancer Research, National Cancer Institute, Bethesda, MD). All the cell lines were cultured as monolayers in Dulbecco's modified Eagle's medium, supplemented with 10% heat-inactivated fetal bovine serum (Hyclone, Logan, UT), 100 µg/ml penicillin and 100 µg/mL streptomycin and maintained in an incubator with 5% CO_2_ at 37°C. Normal human epidermal melanocytes (HEMa-LP, Cat. No. C-024-5C) were obtained from Invitrogen (Carlsbad, CA), and were cultured in HMGS-2 medium supplemented with human melanocyte growth supplement provided by the supplier. For the treatment of cells, silymarin was dissolved in a small amount of acetone, which was added to the complete cell culture medium [maximum concentration of acetone, 0.1% (v/v) in media] prior to addition to subconfluent cells (60–70% confluent). Cells treated with acetone alone served as a vehicle control.

### Chemicals and antibodies

Purified silymarin was purchased from Sigma Chemical Co. (St Louis, MO). The antibodies specific for β-catenin were purchased from R&D Biosystems (Minneapolis, MN), while antibodies for phospho β-catenin, CK1α, GSK-3β, matrix metalloproteinase (MMP)-2, MMP-9, β-transducin repeat-containing proteins (β-TrCP) and β-actin were obtained from Cell Signaling Technology (Beverly, MA). Antibody specific to β-catenin for immunostaining was obtained from R&D Biosystems (Minneapolis, MN). Respective secondary antibodies (rabbit anti-goat and goat anti-rabbit) conjugated with horseradish peroxidase were purchased from Santa Cruz Biotech (Santa Cruz, CA). Boyden Chambers and polycarbonate membranes (8 µm pore size) for cell migration assays were obtained from Neuroprobe (Gaithersburg, MD).

### Cell proliferation assay

The effect of silymarin on the viability of melanoma cells was determined by 3-(4,5-dimethylthiazol-2-yl)-2,5-diphenyltetrazolium bromide assay (Sigma) or MTT assay, as previously described [19]. A total of 1×10^4^ cells per well in 200 µL complete medium were seeded in a 96-well plate and treated with silymarin as previously described [19]. All treatment concentrations were repeated in six wells.

### Matrigel invasion assay

The migration capacity of melanoma cancer cells was determined *in vitro* using Boyden Chambers in which the two chambers were separated with matrigel coated Millipore membranes (6.5 mm diameter filters, 8 µM pore size), as detailed previously [20]. Briefly, melanoma cells (1.5×10^4^ cells/200 µL serum-reduced medium) were placed in the upper chamber of Boyden chambers. Test agents were added to the upper chamber (200 µL) and the lower chamber contained the medium alone (150 µL). Chambers were assembled and kept in an incubator for 24 h or 8 h. At the desired time point, cells from the upper surface of Millipore membranes were removed with gentle swabbing and the migrant cells on the lower surface of membranes were fixed and stained with crystal violet. Membranes were then washed and mounted onto glass slides. The membranes were examined microscopically and cellular migration per sample was determined by counting the number of stained cells in at least four to five randomly selected fields visualized with an Olympus BX41 microscope. Data are presented as mean number of the migrating cells ± SD per microscopic field per sample. Each cell migration experiment was repeated at least three times. Representative photomicrographs were obtained using a Qcolor5 digital camera system fitted to an Olympus BX41 microscope.

### Scratch assay or wound healing assay

Wound healing assay was performed to detect melanoma cell migration, as detailed previously [20]. Briefly, melanoma cells were grown to full confluency in six-well plates and incubated overnight in starvation medium. Cell monolayers were wounded with a sterile 100 µL pipette tip, washed with starvation medium to remove detached cells from the plates. Cells were left either untreated or treated with indicated doses of silymarin in full medium and kept in a CO_2_ incubator for 24 h. After 24 h, medium was replaced with phosphate-buffered saline (PBS) buffer, the wound gap was observed and cells were photographed using an Olympus BX41 microscope fitted with digital camera.

### Immunofluorescent detection of β-catenin

Human melanoma cells (A375 and Hs294t cells) were treated with various concentrations of silymarin (0, 10, 20, and 40 µg/mL) for the desired time period. The cells were then harvested and processed for cytospin preparation (1×10^5^ cells/slide) for immunofluorescent staining and detection of nuclear β-catenin. Briefly, cells were fixed with methanol at −20°C for 10 minutes and non- specific binding sites were blocked with 2% bovine serum albumin (Sigma, St Louis, MO) in PBS for 30 min. Cells were permeabilized with 0.2% Triton X-100 (Sigma Co., St. Louis, MO) in PBS and then incubated with β-catenin-specific antibody for 2 h at room temperature. The cells were washed with PBS buffer and β-catenin was detected by an Alexa fluor 594-conjugated secondary antibody. Cells were mounted with Vectashield mounting medium for fluorescence and stained with DAPI (Vector Laboratories, Burlingame, CA) before they were observed with a fluorescence detection equipped microscope and photographed.

### Immunoprecipitation and immunoblotting

Following treatment of melanoma cells with or without silymarin or other agents for the indicated time periods, the cells were harvested, washed with cold PBS buffer and lysed with ice-cold lysis buffer supplemented with protease inhibitors, as detailed previously [20]. Nuclear and cytosolic fractions were also prepared from the cells of different treatment groups following standard protocols, as described earlier [20]. Equal amounts of proteins from each treatment group were resolved on 10% Tris/Glycine gels and transferred onto a nitrocellulose membrane. After blocking the non-specific binding sites, the membrane was incubated with the primary antibody at 4°C overnight. The membrane was then incubated with the appropriate peroxidase-conjugated secondary antibody and the immunoreactive bands were visualized using the enhanced chemiluminescence reagents. To verify equal protein loading, the membrane was stripped and re-probed with anti-β actin antibody. Each experiment was repeated at least three times for western blotting and representative blots are presented.

For β-TrCP binding assay, A375 melanoma cells were treated with vehicle or various concentrations of silymarin for 24 h, washed with ice-cold PBS, and whole cell lysates prepared as described previously [20]. Aliquots containing 200 µg of protein were cleared with protein A/G-plus agarose beads (Santa Cruz, CA). β-TrCP protein was immunoprecipitated from whole cell lysates by overnight incubation with anti-β-TrCP antibody at 4°C followed by the addition of protein A/G-plus agarose beads (50 µL, Santa Cruz, CA) and continued incubation for 2 h. Immunoprecipitates were washed, and subsequently subjected to SDS-PAGE on 10% gels followed by immunoblotting using antibodies specific to phospho forms of β-catenin.

### Statistical analysis

For migration assays, the control and silymarin-treatment groups were compared using one-way analysis of variance (ANOVA) followed by *post hoc* Dunn's test using GraphPad Prism version 4.00 for Windows, GraphPad Software, San Diego, California, USA, www.graphpad.com. All quantitative data for cell migration are shown as mean ± SD/microscopic field, and each experiment was repeated at least 3 times. In each case *P*<0.05 was considered statistically significant.

## Results

### Comparative migratory behavior of human melanoma cells and normal human epidermal melanocytes

First the studies were performed to examine the migratory behavior of melanoma cells and normal human epidermal melanocytes under identical conditions. For this purpose, cells were kept in Boyden chambers for invasion assays for 24 h in an incubator to assess their migration capability. As shown in Figure 1A, the cell migration capacity of melanoma cells was significantly higher (*P*<0.001) than normal human epidermal melanocytes. The migration of A375 cells was greater than Hs294t cells (390±14 cells/microscopic field for A375 vs 340±12 cells/microscopic field for Hs294t). Under identical conditions, migration of normal human epidermal melanocytes was significantly lower (19±4 cells per microscopic field, *P*<0.001) than melanoma cells, as summarized in Figure 1B.

**Figure 1:** Migration ability of human melanoma cells and normal human epidermal melanocytes. (A) Equal numbers of human melanoma cells (A375 and Hs294t) and normal human epidermal melanocytes (HEMa) were subjected to cell migration by standard invasion assay using Boyden chambers. Twenty four h later, migratory cells were detected on the membrane after staining the migratory cells with the 0.1% crystal violet dye. Representative photomicrographs are shown from three independent experiments. (B) The migratory cells were counted and the results expressed as the mean number of migratory cells ± SD per microscopic field (n = 3). Significantly less migration of normal human melanocytes *versus* melanoma cells, ^*^ *P*<0.001. (C) Chemical structure of silibinin, the major and most biological active component of silymarin.

### Silymarin inhibits human melanoma cell migration: wound healing assay

Molecular structure of silibinin is shown in Figure 1C, which is a major (90%) and most active component of silymarin. We first determined whether treatment of A375 and Hs294t human melanoma cells with silymarin inhibited their migration using a wound healing assay, as described in Material and Methods. Before conducting this assay, preliminary screening experiments were performed to determine the effects of lower (low, non-death-inducing) concentrations of silymarin (0–40 µg/mL) that did not induce cell death in melanoma cells. As shown in Figure 2A, relative to untreated control cells, treatment of cells with various concentrations of silymarin (0, 10, 20 and 40 µg/mL) reduced the migration capacity of A375 and Hs294t cells in a concentration-dependent manner after the treatment of cells for 24 h. The major part of gap or wounding space between cell layers after making a wound was occupied by the migrating A375 cells which were not treated with silymarin. However, the healing of the wound or the empty space of the cells was largely not occupied by the migrating cells treated with silymarin and this effect was dose-dependent. The gap or wounding space between the cells is highlighted by broken red lines, as shown in Figure 2A. These observations suggest that silymarin inhibited the migration of melanoma cells. To confirm that the inhibition of cancer cell migration by silymarin was a direct effect on cell migration and not due to a reduction in cell viability, a trypan blue assay was performed using cells that were treated identically to those used in the migration assays. Treatment of A375 and Hs294t cells with various concentrations of silymarin (0, 10, 20 and 40 µg/mL) for 24 h had no significant effect on cell viability or cell death (data not shown).

**Figure 2:** Silymarin inhibits melanoma cell migration and/or invasion in a concentration-dependent manner. (A) Wound healing assay was performed to assess the effect of silymarin on the migration of A375 and Hs294t human melanoma cells. Incubation of A375 or Hs294t cells with silymarin for 24 h inhibits migration of cells in a concentration-dependent manner compared to non-silymarin-treated control cells. Broken red line indicates the gap without the presence of cells. Assay was repeated three times and representative pictures are shown. (B) Treatment of human melanoma cells with silymarin inhibits migration or invasion ability of cells. Treatment of A375 or Hs294t human melanoma cells with silymarin for 24 h inhibits invasion of cells in a concentration dependent manner. (C) The migratory cells were counted on membrane in at least four to five randomly selected microscopic fields and the results are summarized and expressed as the mean number of migratory cells ± SD per microscopic field. Significant difference *versus* non-silymarin treated control group, ^*^ *P*<0.001, ^**^ *P*<0.01.

### Silymarin inhibits melanoma cell invasion: Boyden chamber assay

Since cell invasion is a key step involved in tumor metastasis, inhibition of cell invasion by the use of phytochemicals, such as silymarin, may represent an important strategy to prevent melanoma metastasis. Therefore, we determined whether treatment of A375 and Hs294t human melanoma cells with silymarin inhibited their invasive potential using Boyden chamber cell invasion assay. Again, preliminary screening experiments were performed to determine the effects of lower concentrations of silymarin that did not induce melanoma cell death (data not shown). As shown in Figure 2B, relative to untreated control cells, treatment with silymarin at concentrations of 10, 20 and 40 µg/mL reduced the migratory capacity of A375 and Hs294t cells in a concentration-dependent manner. The density of the migrating cells on the membrane after staining with crystal violet is shown in Figure 2B, and the numbers of migrating cells/microscopic field are summarized in Figure 2C. The cell migration was inhibited by 25 to 75% (*P*<0.01−0.001) in A375 cells and by 26–67% (*P*<0.01−0.001) in Hs294t cells in a concentration-dependent manner after treatment with silymarin for 24 h.

### Silymarin reduces nuclear accumulation of β-catenin

Activation of β-catenin has been implicated in cancer cell migration. Therefore, we determined the effect of silymarin on the levels of β-catenin protein on both A375 and Hs294t cells using western blot analysis. For this purpose cells were treated with silymarin for 24 h and whole cell lysates, cytosolic and nuclear fractions were prepared. Western blot analysis revealed that treatment of A375 and Hs294t cells with silymarin for 24 h resulted in reduction of β-catenin levels in the nucleus of the cells (Figures 3A and 3D). This change correlated with an increase in cytosolic β-catenin. These observations were further checked and verified in melanoma cells using immunofluorescence staining (Figures 3C and 3F). Magnified cells inside the box clearly show the reduced staining of nuclear β-catenin after the treatment of cells with silymarin. As MMP-2 and MMP-9 are the downstream targets of β-catenin [21]–[23], we also measured the effect of silymarin on the levels of MMP-2 and MMP-9. Consistent with the decreased nuclear localization of β-catenin after treating the cells with silymarin, the expression of MMP-2 and MMP-9 were also found to be decreased in both A375 and Hs294t cells after treatment of the cells with silymarin for 24 h (Figures 3A and 3D).

**Figure 3:** Effect of silymarin on β-catenin and its signaling molecules in melanoma cells. (A) Effect of silymarin on the cytosolic and nuclear accumulation of β-catenin, and MMP-2 and MMP-9, which are downstream targets of β-catenin, in *BRAF*-mutated A375 cells. (B) Effect of silymarin on phosphorylation of β-catenin at “critical residues” and on the expression levels of regulatory kinases (GSK-3β, CK1α) implicated in determining nuclear/cytoplasmic accumulation of β-catenin. (C) Immunofluorescence staining shows decrease in nuclear accumulation of β-catenin in A375 cells after the treatment of cells with silymarin for 24 h in a dose-dependent manner. Magnified nuclear staining is shown in the cells inside the box. (D) The effect of silymarin on nuclear and cytosolic levels of β-catenin and its target MMPs proteins important for the cell migration in Hs294t cells after the treatment of cells for 24 h. (E) Effect of silymarin on phosphorylation of β-catenin at “critical residues” and on the expression levels of regulatory kinases (GSK-3β, CK1α) in metastasis-specific Hs294t cells. (F) Immunofluorescence staining showing decrease in nuclear accumulation of β-catenin in Hs294t cells in a dose-dependent manner after treatment of cells with silymarin for 24 h. Magnified nuclear staining is shown in cells inside the box.

Since, nuclear accumulation of β-catenin is inversely correlated with phosphorylation at certain key residues of β-catenin (Ser^45^, Ser^33^, Ser^37^ and Thr^41^), we checked the effect of silymarin on the levels of β-catenin phosphorylation at these sites. Western blot analysis revealed that treatment of A375 and Hs294t cells with silymarin increased the phosphorylation of β-catenin at Ser^45^, and Ser^33^/Ser^37^/Thr^41^ in both melanoma cell lines (Figures 3B and 3E). Further, silymarin treatment of melanoma cells resulted in a dose-dependent increase of CK1α and GSK-3β. Both CK1α and GSK-3β are known to target β-catenin for proteasomal degradation *via* combined phosphorylation at key residues of β-catenin [12].

### Silymarin enhances binding of β-TrCP to phospho forms of β-catenin

It has been shown that β-transducin repeat-containing proteins (β-TrCP) are components of the ubiquitin ligase complex targeting β-catenin for proteasomal degradation and are thus a negative regulator of Wnt/β-catenin signaling [24], [25]. Therefore, we were interested to check whether silymarin has any effect on the expression levels or activity of β-TrCP in our melanoma invasion model. For this purpose, A375 melanoma cells were treated with silymarin for 24 h, cell lysates were prepared, and β-TrCP was immunoprecipitated for detection of its binding with the phospho forms of β-catenin. Western blot analysis data revealed that silymarin did not affect the expression levels of β-TrCP after the treatment of cells for 24 h (data not shown). However, treatment of A375 cells with silymarin enhanced the binding of β-TrCP with phospho forms of β-catenin in a dose-dependent manner, as shown in Figure 4. These data suggest that silymarin may have inactivated β-catenin by enhancing the proteasomal degradation of the β-catenin after its binding with β-TrCP.

**Figure 4:** Treatment of melanoma cells with silymarin enhances binding of β-TrCP with phospho forms of β-catenin. Cells were treated with and without silymarin for 24 h and cell lysates were prepared. In binding assay, β-TrCP was immunoprecipitated using specific antibody from total protein lysates followed by western blot analysis for phospho forms of β-catenin, as detailed in Materials and Methods. IP, immunoprecipitation; IB, immunoblotting.

### Specific activation of β-catenin leads to enhanced cell migration

As we found that silymarin exerts a significant inhibitory effect on the migration of A375 and Hs294t cells, and this inhibition was associated with a decrease in nuclear accumulation of β-catenin in both metastasis-specific melanoma cell lines, next we examined the role of β-catenin in melanoma cell invasion. For this purpose we selected two different melanoma cell lines: one was Mel 1241, which possesses constitutively active Wnt/β-catenin signaling and second one was Mel 1011 (lack activated β-catenin) from which Mel 1241 was derived. First the cell migration ability of these two melanoma cell lines was examined. Our preliminary analysis of cell migration indicated that the cell migration ability of Mel 1241 cells after 24 h was exceptionally higher than A375 or Hs294t cells. Therefore, we reduced the incubation period of the cells to 8 h for subsequent measurement of cell migration using the invasion assay. As shown in Figure 5A, the cell migration activity of Mel 1241 cells after 8 h was significantly higher than the cell migration activity of the Mel 1011 cells. The number of migrating cells of Mel 1241 cells was 499±40 cells/microscopic filed whereas the number of migrating cells of Mel 1011 cells were 29±4 cells/microscopic field, as summarized under Figure 5B (n = 3).

**Figure 5:** Silymarin inhibits human melanoma cell migration by targeting β-catenin. (A), Comparison of invasion ability of two different melanoma cell lines, one has stabilized mutation in β-catenin (Mel 1241) and another possesses wild-type β-catenin (Mel 1011). The migration capacity of Mel 1241 cells after 8 h is significantly higher than the migration capacity of Mel 1011 cells. (B) The migratory cells were counted under microscope and the results are summarized and expressed as the mean number of migratory cells ± SD per microscopic field. Significant difference *versus* Mel 1241 cells, ^*^ *P*<0.001. (C), Treatment of Mel 1241 melanoma cells with silymarin for 8 h inhibits migration of Mel 1241 cells in a concentration dependent manner. (D) The migratory cells were counted under microscope and the results are summarized and expressed as the mean number of migratory cells ± SD/microscopic field (n = 3). Significant inhibition *versus* non-silymarin-treated control, ^*^ *P*<0.001. (E) The effect of silymarin on the Mel 1011 melanoma cell migration after the treatment for 8 h. (F) The migratory cells were counted under microscope in different treatment groups and the results are summarized and expressed as the mean number of migratory cells ± SD/microscopic field (n = 3). Representative photomicrographs of cell migration are shown from three identical experiments.

### Silymarin or FH535, an inhibitor of β-catenin, inhibits melanoma cell invasion ability by targeting β-catenin

To examine whether silymarin inhibits melanoma cell migration by targeting β-catenin, cell migration experiment was conducted with Mel 1241 and Mel 1011 cells with and without the treatment of cells with various concentrations of silymarin (0, 10, 20, and 40 µg/mL) for 8 h. As shown in Figure 5C, treatment of Mel 1241 cells with silymarin significantly inhibited (*P*<0.001) the migration of Mel 1241 cells in a concentration-dependent manner. Resultant cell migration data are summarized in terms of mean number of migrating cells ±SD/microscopic field for different treatment groups in Figure 5D. In contrast, silymarin did not inhibit the cell migrating ability of Mel 1011 cells, which have inactivated β-catenin (Figure 5E). In other words Mel 1011 cells were resistant to the effect of silymarin on their cell migrating behavior. A summary of migrating cells under different treatment groups is shown in Figure 5F.

Further, in support of these observations, Mel 1241 and Mel 1011 cell lines were treated with various concentrations of FH535 (0, 20, 40 and 60 µM) for 8 h and cell migration was analyzed. FH535 has unique ability to inhibit Wnt/β-catenin pathway [26]. As shown in Figure 6A, treatment of Mel 1241 cells with FH535 inhibited the migration of cells in a dose-dependent manner (40–84%, *P*<0.001). Mean number of migrating cells per microscopic field± SD in different treatment groups are summarized in Figure 6B (n = 3). In contrast, FH535 did not inhibit the migration of Mel 1011 cells or Mel 1011 cells were resistant to the effect of FH535 on their cell migrating behavior (Figures 6C, 6D). These data along with the data from silymarin treatment suggest that activation of β-catenin stimulates melanoma cell invasion while its inactivation suppresses the migration of melanoma cells.

**Figure 6:** Effect of FH535, an inhibitor of β-catenin, on melanoma cell migration. (A) Mel 1241 cells were incubated with FH535 for 8 h and cell migration was determined using invasion assay. FH535 inhibits the cell migration of Mel 1241 cells in a dose-dependent manner. (B) The migratory cells were counted on the membrane under microscope and the results are expressed as the mean number of migratory cells ± SD per microscopic field. Significant inhibition *versus* control, ^*^ *P*<0.001, ^**^ *P*<0.01. (C) Treatment of Mel 1011 cells with FH535 for 8 h did not inhibit cell migration compared to non-FH535-treated control. (D) Migratory cells were counted under microscope and the results are expressed as the mean number of migratory cells± SD per microscopic field. Migration assays were repeated three times and representative pictures of cell migration are shown. No statistical significance of difference *versus* un-treated controls.

In continuation with these studies, the effect of silymarin and FH535 was also determined on the nuclear accumulation of β-catenin, its down-stream targets (MMP-2 and MMP-9) and phosphorylation of β-catenin at various Ser residues using Mel 1241 and Mel 1011 cell lines. For this purpose, cells were treated with and without silymarin or FH535 for 8 h, and cell lysates were prepared for western blot analysis. Western blot analysis revealed that treatment of Mel 1241 cells with both silymarin or FH535 for 8 h resulted in reduced nuclear accumulation of β-catenin and reduced levels of MMP-2 and MMP-9 compared to control cells which were not treated with silymarin or FH535, as shown in Figure 7A. Similarly, the phosphorylation of β-catenin at Ser^45^, and other target residues (Ser^33^/Ser^37^/Thr^41^), and the levels of CK1α and GSK-3β were increased after the treatment of Mel 1241 cells with silymarin or FH535 (Figure 7B). However, these effects of silymarin and FH535 were not observed in Mel 1011 cell line under identical condition (data not shown) or the Mel 1011 melanoma cells were resistant to the action of silymarin and FH535.

**Figure 7:** Effect of silymarin and FH535 on β-catenin and its signaling molecules in Mel 1241 cells. (A) Effect of silymarin and FH535 on the cytosolic and nuclear accumulation of β-catenin, and MMP-2 and MMP-9 in Mel 1241 cells. Cells were treated with silymarin or FH535 for 8 h then harvested, nuclear and cytosolic fractions were prepared and subjected to western blot analysis. (B) Effect of silymarin and FH535 on phosphorylation of β-catenin at “critical residues” and on the expression levels of regulatory kinases (GSK-3β, CK1α) implicated in activation of β-catenin. (C) The combined effect of silymarin and FH535 on Mel 1241 cell migration. Cells were treated with the indicated low doses of silymarin and FH535 either alone or in combination for 8 h and cell migration was determined using invasion assay. Cell migration data are expressed as the mean number of migratory cells ±SD per microscopic field (n = 3). Significant inhibition *versus* untreated control, ^*^ *P*<0.001, ^*^ *P*<0.01. Significant inhibition *versus* either agent alone, ^¶^ *P*<0.01.

### Combined effect of silymarin and FH535 on melanoma cell (Mel 1241) invasion

We further checked the combined effect of silymarin and FH535 on the invasion ability of Mel 1241 cells and this effect was compared with the individual effect of silymarin and FH535 in these cells using identical cell invasion protocol. As shown in Figure 7C, treatment of Mel 1241 cells with low doses of silymarin (20 µg/mL) and FH535 (20 µM) separately for 8 h inhibited the cell migration respectively by 54% and 40% compared to non-treated control cells. However, the invasion activity of Mel 1241 cells was significantly inhibited (81%, *P*<0.01) when the cells were treated with silymarin plus FH535 compared with either agent alone, as shown in Figure 7C.

## Discussion

The significant findings of the present study are that silymarin inhibits invasion or cell migration ability of melanoma cells in a dose-dependent manner, and that is associated with the inactivation of β-catenin signaling pathway. Based on our observation, cells will go under apoptosis or cell death if melanoma cells are treated with silymarin for more than 24 h time period or at a higher concentration of silymarin (>40 µg/mL). Under these conditions, cell migration will decrease, and this reduction in cell migration could be due to reduced cell viability or cell death and not because of changes in migrating behavior of cells. In our study, cell death or apoptosis is not a reason of silymarin-caused inhibition of melanoma cell migration. Silymarin has been shown to inhibit skin carcinogenesis [4]–[6], and has pleiotropic activities which include the inhibition of cyclooxygenase-2 (COX-2) activity and an inhibitor of polyamine biosynthesis [4], [5]. Traditional non-steroidal anti-inflammatory drugs (NSAIDs), such as sulindac, inhibit COX-2 expression resulting in reduced Wnt-signaling by induced β-catenin degradation, as has been shown in colon cancer [27]. Similar to the function of NSAIDs, silymarin also induced β-catenin degradation in melanoma cells and that is associated with inhibition of melanoma cell migration.

Various studies have implicated the role of constitutively active Wnt/β-catenin signaling in tumor progression. β-catenin is a dual function protein and is an important component of cell-cell adhesion, where it forms a dynamic link between E-cadherin and cytoskeleton [28], [29]. This cell-to-cell adhesion may prevent the migration of cells. However, the breaking of cell-to-cell adhesion due to activation of β-catenin and its nuclear accumulation may increase the migration potential of tumor cells. It can also regulate cell migration via its role as a transcription factor wherein it along with transcription factors of the T-cell factor and lymphoid enhancer factor family regulates expression of various target genes that mediate cellular processes including cell migration [11]. Thus nuclear/cytoplasmic ratio of β-catenin in the cells determines their migration potential. Our results show that silymarin inhibits melanoma cell migration by targeting β-catenin. It has been shown that phosphorylation of β-catenin at critical target residues such as at Ser^45^, Ser^33/37^ and Thr^41^ by GSK-3β and CK1α within the cytosolic destruction complex leads to degradation of β-catenin and thus reduces its nuclear accumulation [12]. In our study, we found that treatment of melanoma cells with silymarin enhances the expression of GSK-3β and CK1α, and β-catenin is phosphorylated at critical target residues. This suggests that silymarin via enhanced expression of GSK-3β and CK1α leads to enhanced phosphorylation of β-catenin at critical residues. This then lead to degradation of β-catenin within the degradation complex resulting in its reduced nuclear accumulation. It thus explains inhibitory effects of silymarin against melanoma cell migration.

Diverse molecular events are integrated in the progression and metastasis of cancer cells. In tumor cells, mechanisms that inhibit GSK-3β-induced phosphorylation of β-catenin block its interaction with the E3 ubiquitin ligase receptor, β-TrCP, which prevents β-catenin ubiquitination and degradation, and ultimately leads to β-catenin activation [24], [25]. Oncogenic activation of β-catenin occurs primarily as a consequence of its stabilization by escaping ubiquitin-mediated proteasomal degradation. A major regulator of β-catenin stability and activity is the β-TrCP. In this study, we sought to determine whether the inactivation of β-catenin in melanoma cells by silymarin is affected by expression of its regulator, the β-TrCP. We found that silymarin enhanced the binding of β-TrCP to phospho forms of β-catenin, which suggests β-TrCP-mediated ubiquitination and degradation/inactivation of β-catenin [25], [30]. Thus, this finding further supports our hypothesis that silymarin inhibits melanoma cell migration by targeting β-catenin.

In an attempt to further verify the role of silymarin on prevention of invasive potential of melanoma cell through inactivation of β-catenin signaling, we used two distinct melanoma cell lines, namely Mel 1241 and Mel 1011. The two cell lines differ in status of constitutive activation of Wnt/β-catenin signaling. Our preliminary data show that Mel 1241 melanoma cells which possess constitutively active Wnt/β-catenin are highly invasive and the capacity of cell migration is multiple-fold higher than A375 and Hs294t cell lines. Treatment of Mel 1241 cells with silymarin resulted in significant inhibition of cell migration which was associated with the reduction in nuclear accumulation of β-catenin and reduction in the levels of MMP-2 and MMP-9 which are the down-stream targets of β-catenin signaling. These observations were supported when treatment of these cells with FH535, an inhibitor β-catenin, also resulted in significant inhibition of Mel 1241 cell migration concomitantly reduced accumulation of nuclear β-catenin and lowering the levels of MMPs. Both silymarin and FH535 elevated the levels of GSK-3β and CK1α and simultaneously enhances the phosphorylation of β-catenin at specific target residues (*e.g.*, Ser^45^, Ser^33/37^ and Thr^41^). Both CK1α and GSK-3β are known to target β-catenin for proteasomal degradation via combined phosphorylation at key residues of β-catenin [12]. Interestingly, under identical experimental conditions, these effects of silymarin and FH535 were not found in the Mel 1011 cell line, which lacks constitutively active β-catenin. Wnt signaling is suggested to inhibit β-catenin phosphorylation, thus inducing the accumulation of cytosolic β-catenin, which associates with the T cell factor/lymphocyte enhancer factor family of transcription factors to activate Wnt/β-catenin-responsive genes [31], [32]. Our study provide evidence that silymarin induced β-catenin phosphorylation degradation in melanoma cells is associated with the up-regulation of CK1α and GSK-3β. Liu et al. [12] have identified CK1α as an essential component that controls β-catenin phosphorylation degradation in *Drosophila*.

In summary, the outcome of this study suggests that silymarin has the ability to block or inhibit the invasive potential of melanoma cells, and this anti-invasion effect of silymarin is mediated through inactivation of β-catenin, as summarized under Figure 8. Thus intervention strategies targeting key molecules of the Wnt/β-catenin pathway may represent promising approaches to inhibit metastasis of melanoma cells. This new insight into the anti-melanoma cell migration activity of silymarin could serve as the basis for chemoprevention or therapy of malignant melanoma in high risk individuals.

**Figure 8:** Schematic diagram depicts the mechanism of inactivation of β-catenin by silymarin in melanoma cells. Silymarin blocks β-catenin activation through stimulation of its phosphorylation at different Serine sites and binding with β-TrCP, which subsequently decreases its nuclear accumulation and that results in inhibition of invasive potential of melanoma cells.
